# Antioxidant and Anticancer Potentials of the Olive and Sesame Mixture against Dimethylhydrazine-Induced Colorectal Cancer in Wistar Rats

**DOI:** 10.1155/2022/5440773

**Published:** 2022-10-10

**Authors:** Amirhasan Valaei, Fatemeh Azadeh, Seyedeh Talayeh Mostafavi Niaki, Alireza Salehi, Maede Shakib Khoob, Seyed Hesam odin Mirebrahimi, Sohrab Kazemi, Seyed Mohammad Hosseini

**Affiliations:** ^1^Department of Pathology, Babol Branch, Islamic Azad University, Babol, Iran; ^2^Cellular and Molecular Biology Research Center, Health Research Institute, Babol University of Medical Sciences, Babol, Iran

## Abstract

Cancer is one of the leading causes of death worldwide, and natural agents have shown some promise in fighting it. Thus, the present study tried to evaluate the healing potential of an equal combination of olive and sesame extract (MOS) against the colorectal cancerous lesions that were induced by dimethylhydrazine (DMH) in male rats and also compare the anticarcinogenic potential of the MOS and vitamin E with each other. Therefore, the mixture of equal olive and sesame extract (MOS) was used as the main treatment, alongside vitamin E as a parallel treatment. This study examined the red blood cell (RBC) and white blood cell (WBC) levels, biochemical indices, lactate dehydrogenase (LDH), C-reactive protein (CRP), total protein (TP), creatine kinase (CPK), albumin, and the colon tissue pathology, as well as the level of protein expression of the adenomatous polyposis coli (APC), proliferating cell nuclear antigen (PCNA), carcinoembryonic antigen (CEA), and platelet-derived growth factor (PDGF). Also, the tissue stress markers including total antioxidant capacity (TAC), malondialdehyde (MDA), and superoxide dismutase (SOD) were analyzed. Overall, the results represented a significant reduction in the congestion, mitotic index, inflammation, and cell destruction in the MOS group compared to the DMH group. In terms of the oxidative stress level, a significant increase was observed in the DMH group in comparison with the DMH-MOS group (*P* < 0.05), and the MOS significantly increased TAC level (*P* < 0.05). Furthermore, the DMH+MOS-exposed group exhibited a significantly lower expression of the PCNA, CEA, and PDGF proteins than those of the DMH group. Overall, the MOS showed that it can effectively prevent DMH-induced colon lesions. This mixture, as a strong antioxidant agent, can be clinically applied for preventing and treating colorectal cancer, the effectiveness of which is higher than that of vitamin E.

## 1. Introduction

Cancer is known among the major causes of mortality and morbidity worldwide [1]. For example, 147950 new cases of colorectal cancer had been reported in the United States over the past year [2]. An increase in the reactive oxygen species (ROS) level has a critical role in this cancer development process. Guéraud [3] suggested the effect of high ROS value on the various signaling pathways is related to proliferation, tumor survival, invasion, and metastasis. To modulate the ROS concentration, the body uses different mechanisms such as the antioxidant-based enzymatic system [4]. Grivennikov [5] proposed a close relationship between peptic ulcers, necrosis, and inflammations with the cancers in this organ. Additionally, applying a combination of two or more therapeutic agents for targeting the various cell protective pathways or other causes is considered the cornerstone of modern cancer therapy. The most important advantages of this issue include the consumption of less dose, the overlap of the agent weaknesses, and even synergistic effects of the agents. The combination-therapy mostly contains heavy anticancer and antioxidative potentials to target the antioxidant pathways that lead to fruitful outcomes in cancer therapy [6].

The severity and prognosis of colorectal cancer are determined by using the markers, the most specific one of which is the CEA. The serum CEA level is low, which enhances when adults develop cancer [7]. Further, PCNA, an antigen for proliferating cell nuclei, operates like a DNA clamp as a factor for the DNA polymerase in eukaryotic cells and is necessary for proliferation. Bolton et al. [8] referred to an improvement in the synthesis and expression of the PCNA in the proliferating cells, which defined cell proliferation as a reliable index for examining tumor cell progression [9]. The absence of APC protein due to chromosomal instability results in forming a tumor because of its role as a brake in the cell divisions [10]. In addition, the expression of PDGF leads to an increase in uncontrollable cell growth and tumorigenesis in cancers and tumors [11, 12]. This factor leads to cancer metastasis [13].

The critical aspect of using naturopathy has been reported consistently [14]. These treatments have exhibited huge benefits such as higher efficiency, fewer adverse effects, more drug bioavailability and stability, and proper therapeutic effect with relatively lower doses compared to synthetic drugs [15, 16].

Olive contains a high value of fatty acids and oleic acids, which are innately anticancer [17]. The anticancer mechanism of olive involves the effect of oleic acid and other available antioxidants on the tissue oxidative stress and a change in the apoptosis rate and gene expression of oncogenes [18]. Along with oleic acid, other substances like natural fatty acids, phenols, and squalene are found in olive oil, all of which exhibit protective properties [19–21].

The results of the previous studies suggested the cancer therapeutic effects of sesame oil [22, 23] and sesame seed [24]. The protective activity of sesame is directly related to its natural antioxidants [25]. The sesame oil or paste can decrease tissue stress [26], and the sesamin is considered the most important anticancer substance in this plant [27].

This study aimed to evaluate the antioxidant and anticancer potentials of the mixture of these two compounds as a single therapeutic agent against colorectal cancer in rats, and compare them with vitamin E, which is a proven anticancer substance [28, 29].

## 2. Method

### 2.1. Extract Preparation

Olive and sesame were freshly obtained from northern Iran (52.35°E and 36.47°N). Sesames were sieved, and olives were separated from their leaves and branches, then were washed, and dried. Then, each compound was individually extracted through indirect aeration under high mechanical pressure, and the oil of which was stored in a refrigerator at 4°C until consumption [30, 31].

### 2.2. Analysis of the Extracts through Employing Gas Chromatography-Mass Spectrometry (GC-MS) Technique

A mixture of olive and sesame oil extracts with equal ratio (MOS) was analyzed by using the GC-MS method to detect its various components (TQ8040 NX, Shimadzu). In this regard, About 1 mL of the mixed extract was injected into the GC-MS using a microsyringe. After comparing the spectra of the constituents with those available in the Wiley and NIST/EPA/NIH34-44 libraries, they were sorted according to the ascending order of their retention time. The relative frequency of each component was reported by stating its maximum level. The values below 1% were removed from the table [32, 33].

### 2.3. Animals

The present study was performed among 60 adult 8 weeks old male Wistar rats, weighing 200-220 g. They were obtained and kept in the animal house of the Pasteur Institute of Iran at 20-23°C in a 12 h light/dark cycle under the relative humidity of 60-70%. It should be noted that the ARRIVE guidelines 2.0 was followed throughout the whole study [34]. Also, this study was approved by the research ethics committees of Islamic Azad University with the approval ID IR.IAU.BABOL.REC.1400.043.

### 2.4. Study Design

Vitamin E and dimethylhydrazine (DMH) were purchased by Merck. Initially, the animals were randomly classified into six groups (10 members).

*Group 1:* the control rats received no treatment, but a normal saline gavage.

*Group 2:* the MOS group received a 1 mL/kg/day dose of the MOS [35] via gavage.

*Group 3:* the vitamin E group received a 180 mg/kg/week dose of vitamin E [36] orally.

*Group 4:* the DMH group received a 30 mg/kg dose of DMH subcutaneously once a week [37, 38].

*Group 5:* the DMH+MOS group received the DMH and MOS simultaneously with the same dose.

*Group 6:* the DMH+vitamin E group was administered the DMH and vitamin E at the same time with the same dose.

After 13 weeks, all rats survived. At the end of the project, for the complete anesthesia, the cocktail of ketamine with10 mg/kg concentration (10%, Bremer Pharma GmbH) and xylazine with 80 mg/kg level (2%, Alfasan Diergeneesmiddelen BV) was applied intraperitoneally injection [39]. Then, the blood and colon tissue samples were gathered, followed by placing two parts of the tissue in formalin and a freezer at -80°C separately for histological assessment and tissue homogenate preparation, respectively.

### 2.5. Blood and Serum Sampling

The blood samples were collected for examining the CBC (Celltac Es MEK-7300 K, Nihon Kohden) and measuring the related serum markers on a BIOLIS24i autoanalyzer (Tokyo Boeki Medisys Inc) [40].

### 2.6. Colon Homogenization

The colon tissue homogenates were utilized by a previously approved method [40]. The homogenates were kept at -80°C until determining the oxidative stress markers.

### 2.7. Oxidative Stress Markers

The levels of MDA, SOD, and TAC in all homogenates were measured by employing the TebPazhouhan Razi, Nasdox, and Naxifer kits, respectively [41]. Regarding each marker, the manual was followed based on the guideline [40].

### 2.8. Western Blot

Similar to the oxidative stress assessment, the homogenates were utilized by the method of a previous study [40]. Further, the primary antibodies of APC, PCNA, CEA, and PDGF (at 4°C for 12 h) and proper secondary antibodies related to peroxidase conjugate were, respectively, applied to incubate the blots. The proportion of antibodies was determined relative to the *β*-actin, which was the control protein. The membranes were rinsed with TBS for 10 minutes and subjected to a PNP-1000D electrophoresis power supply. Finally, the bar indices were analyzed by using the ImageJ software [42, 43].

### 2.9. Histology

For histopathological examination, the colon tissues were placed in a 10% formalin buffer. Then, they were rinsed with normal saline, fixated (DS2080/H, Did Sabz Co.), dehydrated, and passaged to obtain paraffin blocks (TE100, Pouya Abzar Azma). The blocks were cooled (TE100, Pouya Abzar Azma), the five-micron sections of which (DS4055, Did Sabz Co.) were stained with H&E and assessed on an Olympus CX23 optical microscope [44].

### 2.10. Data Analysis

SPSS 26 software, one-way ANOVA, and Duncan's post hoc tests were applied to analyze the data of CBC, serum tests, and stress and inflammatory markers as well as the ratios of western blot proteins. A *P* value less than 0.05 was considered a significant difference. Regarding the histological analysis, the groups were histopathologically scored and a mitotic index was obtained to compare their difference by employing Kruskal-Wallis and Mann–Whitney-*U* assays [44, 45].

### 2.11. Graphical Abstract

To expedite the review by the readers, a graphical abstract has been prepared that briefly depicts the project method and the significant data.

## 3. Results

### 3.1. Analysis of MOS

The results of GC-MS indicated the presence of a great value of oleic acid, palmitic acid, stearic acid, and sesamin in the MOS (Table 1).

### 3.2. Hematological Parameters

Despite the lower RBC, hemoglobin (Hb), RDW, MCHC, MCH, MCV, and hematocrit (HCT) levels in the DMH group had no significant difference observed between the groups (Table 2).

### 3.3. WBC

The results reflected a significant rise and a significant diminution in the total WBC count of the DMH group (*P* < 0.05) and DMH+MOS-receiving (*P* < 0.05) group, respectively. In the DMH group, the neutrophil percentage was elevated, and the lymphocyte percentage decreased significantly (*P* < 0.05), in both of which the MOS improved the WBC ratio (Table 3).

### 3.4. Biochemical and General Serum Inflammatory Markers

Following the use of DMH, the total protein content was enhanced, but it was reduced by receiving the MOS in DMH+MOS group. The groups were not significantly different in terms of the blood albumin level. The DMH groups revealed a significant increase in the LDH and CRP levels (*P* < 0.05) and a rise in the CPK level. All three markers were declined by treating with the MOS significantly (Figure 1).

### 3.5. MDA Level in Colon Tissues

Compared to the control group, the MDA content was significantly elevated in the DMH group (*P* < 0.05), which was diminished among the animals receiving DMH+MOS. Also, a lower level of MDA was seen in the vitamin E group (Figure 2).

### 3.6. SOD Level in Colon Tissues

After exposing the rats to the DMH, a decrease was found in the SOD level compared to the control. However, the MOS-treated group represented a higher SOD level than that of the DMH group (Figure 2).

### 3.7. TAC in Colon Tissues

As displayed in Figure 2, the TAC level was decreased in the DMH group, which significantly was improved in both of the treatment groups (*P* < 0.01) (Figure 2).

### 3.8. Protein Expression Level (Western Blot)

All the protein bands were analyzed (Figure 3). The results indicated a significant reduction in the expression level of APC protein in the DMH group compared to the control group (*P* < 0.05), which then was enhanced by consuming the MOS. The DMH group also showed a significant rise in the expression of CEA protein compared to the control group (*P* < 0.05). Although the CEA level was significantly diminished among the rats exposed to DMH+MOS (*P* < 0.05). In terms of the PCNA protein level, a significant increase was observed in the DMH group compared to the control group (*P* < 0.05), which was significantly decreased in both treatment groups (*P* < 0.05). In addition, a significantly better status was achieved in the animals that received the DMH+MOS than in those which were administrated the DMH+vitamin E (*P* < 0.05). Following the use of DMH, the PDGF protein was significantly more expressed compared to the control group, which was significantly reduced in both treatment groups (*P* < 0.05), while they were not significantly different from the control group (Table 4).

### 3.9. Histological Observations

All of the groups were scored and compared in terms of the characteristic pathological lesions in colon tissue such as the necrosis, mitotic index, and inflammatory cell infiltration level (as the average number of mitoses in 10 HPF at the tumor area, [45]) (Figure 4).

The results demonstrated an insignificant (*P* > 0.05) difference between the control, MOS, and vitamin E-receiving groups regarding necrosis, inflammatory cell, and mitotic levels (Figure 4). However, all three indices of the DMH group were significantly different from those of the first three groups (*P* < 0.05). After scoring and staging, a significant decline was obtained in the necrosis, inflammatory cell infiltration, and mitosis of the DMH+MOS-exposed group compared to the DMH one (*P* < 0.05) (Table 5).

## 4. Discussion

The results of the present study represented a diminution in the anti-inflammatory and anticancer activity in the DMH-exposed colorectal tissue during the carcinogenesis and tumorigenesis phases following the simultaneous administration of the DMH, as well as an equal combination of the sesame and olive oil extracts. The tissue stress and inflammation in the precancerous stage were reduced after using the MOS. This mixture resulted in expressing significantly lower CEA, PCNA, and PDGF proteins (*P* < 0.05) and influenced the blood and serum factors positively. The Wistar rats did not have pseudopoisoning effects because of administering the MOS. DMH is a poisonous substance with carcinogenic and methylation properties, which can lead to various levels of inflammation and precancerous and cancerous lesions [46–48]. The consumption of this compound causes serious lesions in the abdominal tissues, especially the colon [49]. The DMH exerts its effects by damaging the mucus, methylating the tissue, and forming free radicals [50]. In addition, it is shown that oral antioxidants can decline the effects and lesions caused by DMH [51, 52].

The intended oily mixture in this study contained multiple useful fatty acids and many antioxidants, the most important ones of which were oleic acid, palmitic acid, stearic acid, and sesamin. Oleic acid represents an anticancer and anti-inflammatory activity and prevents tumorigenesis and metastasis. It causes cancer cell apoptosis by enhancing the intracellular ROS value [53]. Harada et al. [54] proposed the antitumor effects of palmitic acid on rats, as well as its ineffectiveness on topoisomerase II despite affecting topoisomerase I and increasing cancer cell apoptosis. Further, this acid inhibits the prostate cancer cells from growing in *in vivo* and *in vitro* conditions [55] and causes breast cancer cell apoptosis [56]. Another fatty acid in the MOS is stearic acid, which exhibited anticancer properties and diminishes the growth of breast cancer cell lines in the previous studies [57, 58]. In the present study, the sesamin with the main source of sesame [59] was used as an anticancer substance, which prevented breast cancer development by increasing the cancer cell apoptosis in previous studies [27, 60]. At the cellular level, Hashim et al. [61] found out that the anticancer effects of virgin olive oil in *in vitro* are due to its high phenolic content.

Based on the results, the RBC and WBC levels rose following the consumption of DMH. Given that the RBC is the first body cell that reacts under unnormal conditions such as stress, the RBC count is considered as one of the first stages of estimating the extent of an anomaly [62]. Other abnormalities and diseases such as cancer occur following the changes to the RBCs [63, 64]. Furthermore, DMH is among the compounds that lead to the free radical formation in the blood and oxidative stress in tissues. Thus, a therapeutic agent should exhibit great antioxidant power to decrease the free radicals for regulating the body's antioxidant balance and inhibiting oxidative stress [65–68]. Regarding the erythrocytes, lipid peroxidation leads to interference [69] and increases the stress that disturbs the immune system [70]. Additionally, the elevated WBC count is known as one of the factors that illustrate tumorigenesis and neoplasm. To fight the cancer cells, the phagocyte and lymphocyte percentages were improved compared to the other WBC due to the higher body's need for these cells [71, 72].

The results of the present study indicated a significant rise in the CRP and LDH levels after the administration of the DMH compared to the control group (*P* < 0.05), which was reduced in the treatment groups. More CRP, as an inflammatory biomarker, after consuming the DMH reflects the body's acute phase. The rats receiving DMH+MOS had less level, reflecting a better status, and a diminution in the tissue inflammation. Regarding the LDH, as an enzyme that is available in the most alive cells, its higher level represents the extensive destructions at the cellular level, which was reduced in this study by utilizing the MOS. The increase in the CPK level can be attributed to skeletal muscle problems, heart damage, and myocardial microinfarction. In this study, the number was elevated due to the DMH-induced liver injury, followed by a decline in the treatment group [73–75].

The three tissue stress markers were significantly increased in the DMH group compared to the control group (*P* < 0.05). Moreover, the histological observations of colon revealed the necrotic and inflammatory lesions. The DMH group experienced a decline in the SOD content (an antioxidant enzyme) compared to the control group [76]. High lipid peroxidation level in the colon tissue is directly related to the severity of DMH-induced lesions [77]. Lipid peroxidation products are considered the oxidative stress biomarkers to specify the extent of cell injury [78]. In this regard, a significantly greater MDA concentration was seen in the DMH group compared to the control group (*P* < 0.05), which is a tissue stress index. In addition to leading to oxidative stress, lipid peroxidation products also represent the necrotizing effects and increase the neoplasm rate [79]. A rise in the MDA or a decrease in the TAC level following the administration of a DMH reduces the body's ability to fight oxidative stress and exacerbated peroxidation-caused lesions. Also, the MOS with a high antioxidant activity significantly elevated the TAC level in the treatment group compared to the DMH group (*P* < 0.05) and promoted the power of the body's antioxidant system against the free radicals and metabolites that were formed in the lipid peroxidation cycle. The TAC level and metabolites that are created during the oxidation process (MDA) can be used to calculate the level of tissue's oxidative stress [80, 81]. According to Favoriti et al. [82], a more accurate prognosis can be obtained by considering the pathological assessment and some serum markers, as the general indices of inflammation and cell injuries.

The expression levels of the APC, PCNA, CEA, and PDGE proteins in the tissue were assessed relative to the *β*-actin protein [83]. The results demonstrated a significantly higher CEA expression in the DMH group compared to the control group (*P* < 0.05), which reflected the cancerous status of that tissue. CEA content is often enhanced by the tumor cell secretions. In this study, the CEA level was risen in the colon tissue due to the effect of the DMH on this tissue, as well as disruption in its oxidant balance and the following methylation and mutation. The main reason for that rise in protein concentration was the probable presence of cancerous cells in the colon tissue. Compared to the control group, this content was significantly reduced in the DMH+MOS group because of the establishing oxidant balance in this tissue (By another mean, removing the initial cause of the carcinogenesis cascade of the DMH). The PCNA protein had more expression in all cancerous tissues following the use of DMH in comparison with the control group. The results indicated the antiproliferative properties of the MOS on cells, particularly cancer cells. It represented an anticancer effect by inhibiting the cells from proliferating. Regarding the APC level, the DMH group experienced a significant decrease compared to the control group (*P* < 0.05), and elevated unbridled cell divisions and tumorigenesis were observed due to the loss of chromosomal stability. After consuming the MOS, this protein's concentration was improved in cells because of the reexpression of the APC genes, and as a result, the chromosomal stability was enhanced, which caused a controlled cell reproduction cycle and a declined carcinogenesis rate. At last, a significantly greater PDGF level was observed in the DMH group than that of the control group (*P* < 0.05), which was significantly diminished among the rats that were exposed to the DMH+MOS. This result may be ascribed to the inhibition of the factor from production, which was clinically manifested as reduced congestion in histology and less PDGF content in the colon tissue [84].

Finally, based on the results of the histopathological assessment, the different tissue lesions were generated in the Wistar rat colon after using the DMH, which was similar to the results of a previous study. [85]. The lesions were scored and were staged between the groups by using the protocols that were presented by the previous studies [44, 86, 87], the results of which revealed the signs of congestion, necrosis, higher mitotic index, and inflammatory cell infiltration in the DMH-treated rats due to the methylation and an increased in the free radicals of the tissue (Table 5) [88]. In the DMH+MOS group, a significantly lower mitotic index, cell necrosis, and inflammatory cells were observed compared to the DMH group due to the fewer free radicals, because the lipid peroxidation was decreased in the colon tissue (*P* < 0.05). It could be seen that the results of this study are consistent with the results of the previous studies in terms of pathological changes [44, 86, 87].

## 5. Conclusion

Due to the high anti-inflammatory, anticancer, antitumor, and antioxidant activities of the mixture of an equal olive and sesame extract, it is suggested that the administration of this mixture with the 1 mL/kg/daily dose will decrease the oxidative stress by controlling the lipid peroxidation pathway. This mixture declines the free radicals by improving the body's antioxidant defense system substantially. Overall, it controls the cell division markers, which leads to a lower uncontrollable cell division and a diminution in the rate and extent of carcinogenesis and tumorigenesis.

## Figures and Tables

**Figure 1:** Comparison between general serum biochemical indices. ^∗^*P* < 0.05, ^∗∗^*P* < 0.01, ^∗∗∗^*P* < 0.001, and ^∗∗∗∗^*P* < 0.0001: significant compared to the DMH group. All results are expressed as the mean ± standard error. *N* = 10.

**Figure 2:** Comparison between MDA, SOD, and TAC levels in the colon tissue of different groups. ^∗^*P* < 0.05, ^∗∗^*P* < 0.01, ^∗∗∗^*P* < 0.001, and ^∗∗∗∗^*P* < 0.0001: significant compared to the DMH group. All results are expressed as the mean ± standard error. N =6.

**Figure 3:** Western blot bands in grayscale.

**Figure 4:** Comparison of colon tissue indices of the different groups. Normal tissue conditions in the control, MOS (combination oil), and vitamin E groups. Mitosis, necrosis, and inflammatory cells are demonstrated with upward arrows, right arrows, and ^∗^, respectively, in 40× magnification and H&E staining.

**Table 1:** Results of analyzing MOS through GC-MS. Retention time: the time from when the injection was made (initial time) to when elution occurred is referred to as the retention time.

Chemical constituents	Retention time	Peak area (%)	Molecular weight (mg/Mol)	Molecular formula
Palmitic acid	18.503	7.93	256.42	C_16_H_32_O_2_
Oleic acid	20.299	51.58	282.46	C_18_H_34_O_2_
Stearic acid	20.403	5.25	284.47	C_18_H_36_O_2_
Squalene	25.347	7.35	410.73	C_30_H_50_
Stigmastan-3,5-diene	26.715	7.85	396.7	C_29_H_48_
(+)-Sesamin	29.447	11.48	354.35	C_20_H_18_O_6_

**Table 2:** Comparison between RBC parameters. All results are expressed as the mean ± standard error. *N* = 10.

Groups	RBC (×10^6^/*μ*L)	HGB (g/dL)	HCT (%)	MCV (fL)	MCH (pg)	MCHC (g/dL)	RDW (%)
Control	8.12 ± 0.22	13.64 ± 0.45	40.7 ± 1.46	51.06 ± 0.78	17.16 ± 0.34	33.56 ± 0.24	14.35 ± 0.35
MOS	7.85 ± 0.21	13.33 ± 0.29	39.36 ± 1.17	50.58 ± 0.9	17.13 ± 0.14	33.65 ± 0.34	13.53 ± 0.18
Vit E	8.32 ± 0.19	14.15 ± 0.27	41.2 ± 2.04	50.24 ± 0.5	17.08 ± 0.35	33.6 ± 0.48	13.76 ± 0.32
DMH	7.54 ± 0.37	12.94 ± 0.47	39.19 ± 1.78	49.43 ± 1.68	16.99 ± 0.29	32.44 ± 0.33	13.51 ± 0.31
DMH+MOS	7.76 ± 0.22	13.32 ± 0.38	40.25 ± 1.12	49.76 ± 1.32	17.14 ± 0.13	33.06 ± 0.25	13.4 ± 0.3
DMH+vit E	8.09 ± 0.24	13.24 ± 0.4	39.88 ± 1.55	49.51 ± 0.87	17.11 ± 0.24	33.59 ± 0.64	13.61 ± 0.39

**Table 3:** Comparison between platelet and WBC and parameters. ^∗^*P* < 0.05: significant compared to the DMH group. All results are expressed as the mean ± standard error. *N* = 10.

Groups	WBC (×10^3^/*μ*L)	Neutrophil (%)	Lymphocyte (%)	PLT (×10^3^/*μ*L)
Control	7.93 ± 0.44^∗^	59.08 ± 3^∗^	45 ± 3.59^∗^	734 ± 23.84
MOS	7.4 ± 0.33^∗^	57.6 ± 3.16^∗^	41.88 ± 2.99^∗^	722.25 ± 31.09
Vitamin E	7.6 ± 0.48^∗^	62.16 ± 3.64	43.46 ± 2.49^∗^	791.13 ± 23.13
DMH	9.58 ± 0.75	72.4 ± 5.05	26.93 ± 2.96	786.63 ± 51.79
DMH+MOS	7.76 ± 0.51^∗^	60.54 ± 3.99^∗^	37.89 ± 4.12^∗^	788 ± 40.46
DMH+vitamin E	8.2 ± 0.48	70.53 ± 3.18	29.71 ± 2.76	803.63 ± 32.88

**Table 4:** Comparison between the expression level of proteins relative to that of *β*-actin in colon tissue. ^∗^*P* < 0.05: significant compared to the DMH group. All results are expressed as the mean ± standard error. *N* = 6.

Groups	APC	CEA	PCNA	PDGF
Control	0.99 ± 0.02^∗^	0.39 ± 0.01^∗^	0.72 ± 0.03^∗^	0.89 ± 0.0^∗^
DMH	0.65 ± 0.06	0.82 ± 0.09	1.49 ± 0.07	1.38 ± 0.05
DMH+MOS	0.80 ± 0.05	0.46 ± 0.04^∗^	0.75 ± 0.03^∗^	0.94 ± 0.04^∗^
DMH+vitamin E	0.68 ± 0.05	0.71 ± 0.04	1.02 ± 0.05^∗^	0.98 ± 0.11^∗^

**Table 5:** Comparison between the tissue inflammation, mitotic, and necrosis indices of the different groups. *P* values less than 0.0001 were considered statistically significant. All results are expressed as the mean ± standard error. ^a^Statistically significant differences were found between the control and DMH groups. ^b^Statistically significant differences were found between the control and DMH+vitamin E-treated groups. ^c^Statistically significant differences were found between the DMH and DMH+MOS-treated groups. ^d^Statistically significant differences were found between the DMH and DMH+vitamin E-treated groups. *N* = 10.

Groups	Necrosis	Inflammatory cells infiltration	Mitosis
Control	0.20 ± 0.13	0.10 ± 0.10	0.30 ± 0.15
MOS	0.20 ± 0.13	0.20 ± 0.13	0.10 ± 0.10
Vitamin E	0.10 ± 0.10	0.10 ± 0.10	0.20 ± 0.13
DMH	2.10 ± 0.23^a^	1.90 ± 0.28^a^	20.70 ± 1.08^a^
DMH+MOS	1.50 ± 0.22^c^	1.70 ± 0.26^c^	18.20 ± 1.3^c^
DMH+vitamin E	1.20 ± 0.24^b,d^	1.30 ± 0.30^b^	16.70 ± 1.21^b,d^

## Data Availability

The datasets used and analyzed during the current study are available from the corresponding author on reasonable request.
